# Potential Interaction of Fresh Garlic with Metformin during Ischemia-Reperfusion Induced Cardiac Injury in Diabetic Rats

**DOI:** 10.1155/2021/9739089

**Published:** 2021-09-04

**Authors:** Syed Mohammed Basheeruddin Asdaq, S. Lokaraja, Abdulhakeem S. Alamri, Walaa F. Alsanie, Majid Alhomrani, Abdulrahman Hadi Almutiri, Sreeharsha Nagaraja, Mohd Imran

**Affiliations:** ^1^Department of Pharmacy Practice, College of Pharmacy, AlMaarefa University, Dariyah, Riyadh 13713, Saudi Arabia; ^2^Department of Pharmacology, Krupanidhi College of Pharmacy, Bangalore 560035, India; ^3^Department of Clinical Laboratory Sciences, The Faculty of Applied Medical Sciences, Taif University, Taif, Saudi Arabia; ^4^Centre of Biomedical Sciences Research (CBSR), Deanship of Scientific Research, Taif University, Taif, Saudi Arabia; ^5^Ministry of Health, Cluster One Riyadh, King Salman Hospital, Riyadh, Saudi Arabia; ^6^Department of Pharmaceutical Sciences, College of Clinical Pharmacy, King Faisal University, Al-Ahsa 31982, Saudi Arabia; ^7^Department of Pharmaceutics, Vidya Siri College of Pharmacy, Off Sarjapura Road, Bengaluru 560 035, Karnataka, India; ^8^Department of Pharmaceutical Chemistry, Faculty of Pharmacy, Northern Border University, Rafha 91911, P.O. BOX 840, Saudi Arabia

## Abstract

**Methods:**

The study was undertaken on both normoglycemic and alloxan (90 mg/kg) induced diabetic Sprague Dawley rats weighing 150–250 g. At the completion of the treatment phase (30 days for garlic, 250 mg/kg, oral; 10 days for MET, 70 mg/kg, oral), rats were anesthetized and mounted on the modified Langendorff's apparatus. IRI was produced by myocardial no-flow global ischemia. Developed tension (DT) and heart rate (HR) were recorded both before and after ischemia. The perfusate was collected to estimate the leakage of cardiac biomarkers (Creatine Kinase-MB: CK-MB and Lactate dehydrogenase: LDH). Hearts were removed from the setup and utilized to prepare heart tissue homogenate (HTH) and histological slides. The endogenous antioxidants, superoxide dismutase (SOD) and catalase (CAT), in addition to oxidative thiobarbituric acid substances (TBS), were estimated in HTH.

**Results:**

The hemodynamic parameters, including percentage recovery in HR and DT, were found significantly higher in animals pretreated with garlic and MET in diabetic rats (DR). Both SOD and CAT enzyme activities increased significantly while TBS levels were reduced in the HTH of animals treated with garlic and MET. The cardiac markers CK-MB and LDH levels also increased in HTH with a corresponding decrease in the perfusate. The histopathological changes in the heart and pancreas demonstrated noticeable protection of the tissues due to pretreatment with garlic and MET. Taken together, these findings advocate that reactive oxygen species derived from hyperglycemia execute an important function in myocardial global IRI; the therapy of garlic homogenate was found to be effective in alleviating these toxic effects.

**Conclusion:**

The combined therapy of MET and garlic provided synergistic cardioprotection, implying that garlic seems to possess promise in lowering toxic parameters by protecting diabetic induced myocardial injury.

## 1. Introduction

Diabetes mellitus (DM), a diverse endocrine illness signified by hyperglycemia, is caused by a deficiency in insulin production, insulin activity, or both. It is among the leading causes of cardiovascular disease, contributing to 80% of all diabetic deaths. Polyuria, polydipsia, weight gain, polyphagia, and impaired eyesight are all indications of hyperglycemia. Cardiovascular disease (CD) mortality is 2–4 times greater in diabetic individuals than in nondiabetic individuals. DM has been linked to the deterioration of heart function. In diabetic patients, many pathogenic mechanisms can cause myocyte injury and dysfunction [1]. Type 1 DM, an autoimmune disease, causes a complete lack of insulin. Insulin deficiency and insulin resistance (IR) are features of type 2 diabetes [2]. Hyperglycemia, which is caused by insulin insufficiency or IR, produces reactive oxygen species (ROS), which is the primary basis of diabetic heart (DH) injury. The heart is vulnerable to ROS damage owing to its low number of free radical scavengers. In DH, oxidative stress (OS) causes improper expression of genes, distorted signal transduction, and modulation of pathways that lead to programmed cardiovascular cell death [3]. Most of the DM-related morbidity and mortality are caused by microvascular and macrovascular diseases. CD or stroke accounts for over 80% of mortality in people with type 2 DM [4]. The results of regular cellular metabolism, ROS, and reactive nitrogen species (RNS) can have either positive or detrimental consequences. ROS has positive effects at low concentrations and plays a physiological function in the host defense system (against infective pathogens) and a variety of cellular signaling events. Overproduction of ROS/RNS and/or a deficit of antioxidant mechanisms cause the damaging consequences of ROS/RNS, also recognized as oxidative/nitrosative stress. Excess ROS may harm cellular DNA, proteins, and lipids, preventing them from performing their functions normally [5]. The OS reduces several antioxidant enzymes in DH because of hyperglycemia. There is strong evidence that DM/hyperglycemia induces OS and that ROS has a role in developing IR, *ß*-cell malfunctioning, and the long-term microvascular/macrovascular consequences of DM [6–9].

Dietary factors have a significant impact on the progression of certain diseases in human, like CD [10]. Garlic has earned a distinct place in several cultures' folklore as a potent preventive and curative agent throughout the last few decades. Garlic (*Allium sativum*), a member of the Alliaceae family, is said to have come from Central Asia. It is used as traditional medicine, as flavoring agent, and as a functional food all over the world to boost physical and cognitive health. Garlic's therapeutic properties in the treatment of various human illnesses and medical problems have been acknowledged for years. Numerous epidemiologic investigations have found that eating habits comprising garlic as a spice are linked to a lower risk of human diseases [11]. Garlic has also been shown to suppress the etiology of CD, in addition to cancer and other age-related chronic disorders [12]. Garlic and its preparations are known to have cardioprotective, antioxidant, antineoplastic, and antibacterial properties and have been used to prevent and manage atherosclerosis, hyperlipidemia, thrombosis, hypertension, and DM [13] worldwide [14]. Garlic homogenate (GH), when taken in moderation, produces endogenous antioxidant activity and reduces oxidative damage by either enhancing endogenous antioxidant synthesis or lowering the formation of oxidants such as oxygen free radicals [13].

Metformin (MET), a biguanide antihyperglycemic drug, is commonly used to treat type 2 DM. It has favorable outcomes for type 2 DM, like weight loss and improved lipid profile/endothelial function because of its antihyperglycemic impact. As a result, MET is given to people who are IR before they develop hyperglycemia [15]. MET slows the progression of DM by lowering liver glucose synthesis and intestinal glucose absorption while increasing peripheral glucose utilization. It also has a variety of lipid-reducing actions. The insulin receptor, glucagon receptor, glucose transporters, and AMP-activated protein kinase (AMPK) are all potential MET targets [16, 17]. MET has been discovered to help in free radical defense and has a significant impact on cells, causing them to produce more insulin [18, 19]. MET has a peripheral impact; therefore, it does not promote insulin release, and it does not cause hyperinsulinemia or IR like other antihyperglycemic medicines. As a result, MET is believed to be a reliable and efficacious medicine to treat type 2 DM, as well as to protect the remaining *ß*-cells from further insulin release induced by hyperglycemia.

Since garlic has antioxidant properties and MET is a cell-protective drug, a synergistic effect of the two may be possible in preventing cardiac muscle damage. Therefore, the intent of this study was to appraise the potential of oral dietary supplementation of garlic in the presence of MET for the prevention of alloxan-induced diabetic rats (DR) using an ischemia-reperfusion experimental model.

## 2. Materials and Methods

### 2.1. Experimental Animals

The experimental protocol was approved by the institution's Animal Ethics Committee. Male Sprague Dawley (SD) rats in a weight range of 150–250 g were kept at standard conditions and unlimited access to food and drink. The animals were kept in an animal house under standard conditions, as directed by the Committee for Control and Supervision of Experiments on Animals (CPCSEA). The experimental protocol was approved by the Institutional Ethical Committee (KCP/IAEC-27/2119). These experiments were conducted in isolated tissues from a perfused heart and were backed up by biochemical and histological data.

### 2.2. Preparation of Raw GH

Garlic bulbs (*Allium sativum*, Liliaceae family) were obtained from single source of garlic field throughout the research study to keep uniformity of its contents. They were peeled, sliced, and ground into paste and a stock solution of 0/1 g/ml [20] was prepared and administered to animals by oral gavage every day within 30 minutes of its preparation.

### 2.3. Apparatus and Chemicals Used

All chemicals and apparatus used in the experiment were procured and purchased from standard companies with the help of genuine suppliers.

### 2.4. Alloxan-Induced Diabetes

Animals were fasted for one day before the experiment and diabetes was induced by a single dose intraperitoneal administration of alloxan 150 mg/kg body weight [21]. The animals from groups V to VIII (diabetic group) were kept on a high-fat diet for eight consecutive weeks before injecting a dose of alloxan [22]. The blood glucose was checked in all animals 72 hours after alloxan dosing and those with a glucose level of more than 300 mg/dl were used in the study.

### 2.5. Experimental Protocol

The cardioprotective role of combined therapy of garlic homogenate (GH) and MET was determined in diabetic and nondiabetic rats. The male SD rats were divided into eight groups consisting of six animals each. Animals in groups I to IV were nondiabetic. Group I was kept as normal control with vehicle treatment for 30 days by oral gavage. Groups II and III were given GH (GH, 250 mg/kg, 30 days) [23] and MET (MET, 70 mg/kg, 10 days) [24], respectively. Group IV received 30 days of GH treatment (250 mg/kg) with the addition of MET (70 mg/kg) in the last 10 days of GH administration. The animals from groups V to VIII were confirmed cases of diabetic animals. Group V was diabetic control, while groups VI and VII received GH and MET, respectively, whereas group VIII animals were given GH and MET. The doses of GH and MET were like normal groups.

### 2.6. Perfusion of Isolated Rat Heart

For the isolated perfused heart, a modified Langendorff's setup was created and used for research. With minor adjustments, animal models of myocardial ischemia and reperfusion were created using the techniques previously described [25]. The rats were anesthetized with a combination of ketamine hydrochloride (75 mg/kg, intraperitoneal) and xylazine (10 mg/kg, intraperitoneal) [26]. The heart was excised from deeply anesthetized animals and mounted on a modified Langendorff setup and perfused with Krebs-Henseleit solution. A displacement transducer was used to measure the contractile force, which was then recorded on a grass electromechanical recorder.

### 2.7. Myocardial Ischemia and Reperfusion

At the end of the initial 15 minutes of perfusion for equilibrium, tracings were recorded for another 15 minutes before subjecting the heart to 15 minutes of global no-flow ischemia. After that, the regular flow rate (5 ml/min) was restored, and perfusion was continued for another 30 minutes. The level of cardioprotection owing to preventive therapy was examined by measuring the developed tension (DT) and heart rate (HR). A thermoregulated chamber kept the heart at 37°C throughout the experiment to avoid hypothermia-induced cardioprotection [26]. None of the trials lasted more than 2 hours, and the experimental preparation remained stable during that period.

### 2.8. Experimental Parameters

Hemodynamic parameters such as HR and DT were recorded both before and after ischemia and percentage recoveries were calculated. The perfusate (perfusing fluid) was collected after ischemia to estimate the CK-MB and LDH activities in the perfusate to determine the extent of damage to the myocardium due to ischemia. HTH was prepared by a method described by Elastner, 1976 [27], to estimate the activities of CK-MB, LDH [28], SOD, CAT, and TBS [29]. Histological slides of the myocardium and pancreas were prepared and stained with hematoxylin and eosin (H-E) transverse stain to study myocardial and pancreatic cell integrity [30].

### 2.9. Statistical Analysis

One-way analysis of variance (ANOVA) was used to determine statistical significance, followed by Dunnett comparison tests using the GraphPad Prism 8.0 computer software kit. The findings were presented as mean ± standard error of mean (SEM), with a *p*˂0.05 significance level considered.

## 3. Results

### 3.1. Effect on Body Weight and Blood Sugar

Table 1 explains the changes in body weight during the eight weeks of a high-fat diet for diabetic groups (groups V to VIII). The animals selected for this study were in a weight range of 200–250 gm. At the end of eight weeks of a high-fat diet, a significant (*P* < 0.001) increase in the body weight of all animals was observed. Similarly, a significantly (*P* < 0.01) elevated blood sugar level was found in animals of all groups at the end of eight weeks of a high-fat diet that was further augmented significantly (*P* < 0.05) 72 hours after administration of alloxan. None of the animals in any group died or were given insulin doses to control blood sugar levels.

### 3.2. Effect on Cardiac Markers

#### 3.2.1. Effect on CK-MB

As indicated in Figure 1, a significant (*P* < 0.01) fall of CK-MB activity was noticed in the perfusate with a concurrent increase in heart tissue homogenate (HTH) in the groups of rats that were given GH when related to the normal control group. The average reading of a group of animals that received combined therapy of GH (30 days) and MET (10 days) showed a significant (*P* < 0.05) elevation of CK-MB activity in HTH in comparison with MET alone and normal control groups. Alloxan-induced diabetic rats exhibited significantly (*P* < 0.01) low CK-MB activity in HTH with greater leakage of the enzyme in the perfusate. Administration of GH and MET demonstrated the best incline of CK-MB activity in HTH with a decline in enzyme leakage in the perfusate when compared to all other diabetic groups.

#### 3.2.2. Effect on LDH

The activities of LDH enzymes in HTH were significantly (*P* < 0.01) high in GH, MET, and GH + MET groups with normal control (Figure 2). The combined therapy of GH and MET presented significantly (*P* < 0.05) better outcomes when related to MET alone. The leakage of LDH enzymes in the perfusate was significantly (P 0.001) elevated in diabetic animals than in normal control animals. However, prior treatment with GH/MET either individually or together produced a significant (*P* < 0.01) improvement in LDH activity in HTH when compared to diabetic animals. Furthermore, when compared with the MET alone group, the release of LDH enzymes in the perfusate was significantly (P 0.05) lower in animals given GH and MET.

### 3.3. Antioxidant and Oxidant Parameters

#### 3.3.1. Effect on Superoxide Dismutase (SOD) and Catalase (CAT)

Thirty days of GH treatment before the experiment caused a significant (*P* < 0.001) increase in SOD and CAT activities when compared to the normal control group. Further, when animals received both GH and MET, they showed significantly higher CAT activity compared to the MET alone group. A significant (*P* < 0.01) depletion of antioxidant activity was noticed in the diabetic control group compared to the normal control. However, administration of GH alone or along with MET significantly increased the SOD and CAT activities in comparison with diabetic control. Among all treated groups in diabetic animals, the combination of GH and MET showed a greater increase in antioxidant activity (Figure 3).

#### 3.3.2. Measurement of Thiobarbituric Acid Substances (TBS)

The proportion of thiobarbituric acid substances (TBS) produced during the decomposition of lipid hydroperoxides was used to measure lipid peroxidation.  Figure 4 shows the distribution of TBS values across different groups in descending order with a cumulative line on the secondary axis as a percentage of the highest value. The highest value of TBS was found in diabetic rats (DR). In the absence of DM-induced generation of oxidative radicals, 30 days of GH administration resulted in the minimum level of TBS, which is even less than the level of TBS found in normal control animals. However, in the presence of alloxan-induced DM, GH administration was not successful enough to keep the similar level of TBS as found in the absence of DM. The addition of MET to GH therapy has shown a better protective effect in preventing free radical formation in the heart tissue when compared to GH or MET alone.

### 3.4. Haemodynamic Parameters

#### 3.4.1. Developed Tension (DT) and Heart Rate (HR)

The percentage recovery in postischemic DT and HR was significantly (*P* < 0.001) increased in animals that were given GH for 0 days when compared to normal control animals (Figure 5). MET administration for 10 days failed to produce a similar significant result. On the contrary, when MET was introduced during the last 10 days of GH (30 days) treatment, significantly (*P* < 0.05) increased recoveries in both hemodynamic parameters were recorded when compared to the MET alone group. Alloxan-induced diabetic animals showed poor recovery in both DT and HR. GH or MET administration either alone or together produced significant (*P* < 0.001) increased postischemic recovery in both parameters when compared to diabetic control.

### 3.5. Histopathological Studies

After fixing the myocardial tissue in paraffin, sections were prepared on glass slides and stained with H&E stain along with acid Schiff reagent to study the histological changes under a light microscope. The developed slide revealed that the toxic diabetic control group had significantly less integrity than the normal control group and the treated group. MET alone did not affect the diabetic group, but, when combined with garlic, the myocardium was found to be significantly intact. Striation loss and neutrophil infiltration were both reduced in the fiber (Figure 6). The DM-induced group had a poor recovery in terms of inflammatory characteristics, whereas the nondiabetic group had better recovery in terms of inflammation and oedema (Figure 7).

## 4. Discussion

In this study, we found that combining the cardioprotective, antioxidant, and antihyperglycemic activities of garlic homogenate (GH) with the biguanide derivative, metformin (MET), defends the myocardium from ischemia-reperfusion injury (IRI) in alloxan-induced diabetic rats. The results also indicate that prophylactic treatment with MET and GH has a synergistic cardioprotective effect as well as a beneficial effect on the pancreas in alloxan diabetic animals. Furthermore, the current data shows that the cardioprotective efficacy of GH at 250 is due to free radical scavenging. Based on functional recovery and LDH released from the heart during reperfusion, data showed that long-term treatment with GH, alone or in combination with MET, before induction of ischemia significantly protects the DH and myocardial function during ischemia-reperfusion.

Type 2 diabetes mellitus (T2DM) is a complicated disease marked by a decrease in insulin function that will follow a decreased release of insulin from *ß* cells (pancreatic *ß*-cell dysfunction). Animal models must replicate the phenotypic and mimic the disease's developmental phase to be similar to humans. Thus, the T2DM model was established by feeding a high-fat diet to induce insulin resistance, followed by an alloxan injection. At the end of 8 weeks of high-fat diet, rats in the diabetic group became obese and only those that developed a blood glucose level of more than 300 mg/dl after alloxan administration were taken up for the study. Alloxan produces cytotoxic ROS, which is involved in the genesis of pancreatic *ß*-cell dysfunction, ischemic heart disease, and lack of endogenous antioxidant defenses [27]. An artificial standard perfusion of an isolated excised rat heart using modified Langendorff's equipment that is reported to be used for evaluating myocardial dysfunction during ischemia was used in this study [31]. The IRI model was used to cause myocardial damage. Ischemia is a type of cardiac impairment caused by an imbalance in the supply/demand of oxygenated blood to the myocardium. With no-flow global ischemia, the IRI was induced [32]. Myocardial ischemia can result in cellular dysfunction and damage, not only during ischemia but also after subsequent reperfusion. In the case of ischemia injury in isolated hearts, reperfusion injury can be reduced to normal levels by changing reperfusion settings or treating with therapies that have both antioxidant and cardioprotective effects on reperfusion injury. In the HTH, a modest dose of GH (250 mg/kg, orally, 30 days) resulted in less enzyme leakage, a lower amount of reactive free radicals, and increased antioxidant activity. This finding suggests that GH has cardioprotective potential due to its antioxidant properties. ROS (superoxide, etc.) are formed in large quantities during IRI, contributing to myocardial dysfunction and severe cell damage [33]. It should also be noted that diabetic cardiomyopathy is usually instigated by a disproportion between oxidants and antioxidant defenses. As a result, prospective antioxidant therapy should employ antioxidants that supplement endogenous antioxidants or promote their synthesis.

Epidemiologic research indicates a contrary relationship concerning garlic consumption and the evolution of CD. Garlic products have been acclaimed worldwide as remedies for the avoidance and control of DM, hypertension, thrombosis, hyperlipidemia, and atherosclerosis [13]. When comparing the diabetic control group with the normal control group and the treated group, we found that Malondialdehyde (MDA) levels, a lipid peroxidation product, and a marker of OS, were significantly higher in the serum. Lipid peroxide (LP) is a significant pathogenic event in myocardial infarction, and the accumulation of LP suggests various stages/complications of the disease [34]. Increased LP levels cause injury to blood vessels, resulting in the aggregation of platelets at the site of injury [35], which is also a factor in DR developing myocardial damage.

Lipid peroxidation is believed to be a critical mechanism of injury that happens during myocardium reperfusion after an ischemia period. Elevated levels of LP in IRI could be credited with lipid buildup in the heart and irretrievable impairment of myocardial membranes. Thiobarbituric acid reactive substance concentration in plasma is an indicator of OS and lipid peroxidation. Elevated TBS levels are linked to an augmented threat of CD. Due to the difficulty of directly measuring liberated ROS due to their instability, TBS, a stable lipid peroxidation end-product, is normally utilized as a marker of ROS creation. Allicin, a molecule existing in garlic, has increased antioxidant activity [36], and the above study found that it kept the level of LP in the heart almost normal when equated to diabetic control.

Because of the presence of thiosulfonate and S-alkyl-substituted cysteine sulfoxide derivatives, garlic possesses a variety of biological roles. The odor of fresh raw garlic (*Allium sativum*) is instigated by the presence of allicin and volatile substances, which are produced by the act of alliinase on allin. When fresh garlic is mashed or chopped, allin (S-alkyl-substituted cysteine sulfoxide) is hydrolyzed by alliinase. The corresponding derivatives of allicin (alkyl alkane thiosulfinates), ammonia, and pyruvic acid are formed in the presence of water [24, 37]. The garlic tissue is damaged while this enzyme is disconnected from its true substrate. Allin is the primary substrate in fresh raw garlic, and allicin is the predominant thiosulfinate generated by the alliinase-catalyzed reaction, accounting for 60–80% of garlic's full thiosulfonate content [38]. When given prophylactically to MET in DR, the biological activity of allicin performs a vital task in keeping the high level of LP near normal. Other sulfur-encompassing compounds found in raw GH include allyl methyl thiosulfonate, *γ*-L-glutamyl-S-alkyl-L-cysteine, 1-propenyl allyl thiosulfonate, and adenosine, all of which have antioxidant and cardioprotective properties, as well as supporting part in the treatment of diabetic myocardial dysfunction.

IRI promotes the generation of ROS and MDA in cardiac tissue homogenates, along with the concomitant reduction of SOD and CAT. During myocardial infarction, superoxides produced at the injury site regulate SOD and CAT, leading to activity decrease and superoxide buildup that harms the myocardium. The decline of endogenous scavengers in the HTH is a risk factor for diabetic myocardium, and preventive treatment of GH and MET has a protective effect. Increased levels of biomarkers like LDH and CK-MB in the perfusate show that diabetic myocardial cells are exposed during IRI due to an inequality in the myocardium between free radicals and free radical scavengers. The number of these biomarkers in excess in the HTH is an indicator of diabetic myocardial cells. Due to the peroxidation of the cardiac membrane by ROS, changes in the permeability of the plasma membrane cause leaking of these cytosolic enzymes into the perfusate. As a result, the presence of these biomarkers in perfusing fluid (perfusate) and the absence of these biomarkers in HTH reveal substantial diabetic myocardial damage [20].

Abnormalities in free fatty acid (FFA) metabolism are a major contributor to aberrant cardiac function, and they can cause glucose oxidation impairment, which can lead to diabetic cardiomyopathy. These deviations are symbolized by an increase in circulating FFAs due to increased adipose tissue lipolysis, in addition to high tissue FFAs due to hydrolysis of augmented myocardial triglyceride stores, which is a crucial risk factor for the initiation and advancement of atherosclerosis and one of the major risk factors in diabetic myocardium in rats. Garlic has antiatherogenic and lipid-lowering properties due to organosulphur compounds that may inactivate the thiol group (-SH) comprising enzymes like 3-hydroxy-3-methyl-glutaryl-coenzyme A (HMG-Co-A) reductase and fatty acid synthase [39]. Earlier research revealed that garlic aqueous extract had an active fraction other than S-allyl cysteine sulfoxide that lowered glucose and cholesterol levels. The component responsible for the antiatherosclerotic action has been identified as allicin [40]. As a result, pretreatment with GH keeps hyperglycemia at a normal level, regulates FFA metabolism, and has a positive effect on pancreatic *ß* cells as well as cardioprotective potential.

Since MET has a peripheral action in type 2 DM, it will reduce hyperglycemia while also assisting GH in lowering hyperinsulinemia levels to normal levels. In type 2 DR, hyperinsulinemia is caused by IR, which stimulates sympathetic activity, causing an increase in Na + reabsorption in the kidneys and an increase in blood pressure, resulting in endothelial dysfunction. When compared to normal rats, our findings from histopathology studies show that the center of islet cells is composed of *ß* cells (70%) with basophilic granules, while the periphery is composed of alpha cells with eosinophilic granules (25%) in the combination treatment, which aids in protecting the *ß* cells from further damage in DR. This study's findings are consistent with another study that found MET to play an imperative role in heart and pancreatic cells [41]. MET not only protects type 2 diabetics from CD and heart failure, but it also restores insulin secretion and protects pancreatic cells from lipotoxicity and glucotoxicity [42, 43]. Furthermore, concomitant treatment of MET with GH enhances their effects and promotes pancreatic cell integrity in addition to myocardial protection.

## 5. Conclusions

In this study, the prophylactic administration of garlic homogenate with the antidiabetic and cardioprotective synthetic drug metformin helped protect the isolated diabetic heart during ischemic reperfusion injury. Moreover, garlic homogenate in combinational therapy decreases pancreatic oxidative radical increase and promotes the antioxidant defense system, correcting hyperinsulinemia and *ß*-cell viability in alloxan-induced diabetic rats.

## Figures and Tables

**Figure 1:** Effect on CK-MB activity. Data are given as mean ±SEM, where ^∗∗^*P* < 0.001, compared to normal control; ^•••^*P* < 0.001, compared to diabetic control; °P <0.05 and °°P <0.01, compared to MET; N-GH, normal-GH of 250 mg/kg; N-MET, normal-MET of 70 mg/kg; N-(GH + MET), GH plus MET in normal rats; D-GH, GH of 250 mg/kg in diabetic rats; D-MET, MET of 70 mg/kg in diabetic rats; and D-(GH + MET), GH plus MET in diabetic rats.

**Figure 2:** Effect on LDH activity. Data are given as mean ±SEM, where ^∗∗^*P* < 0.01 <0.01 and ^∗∗∗^*P* < 0.001, compared to normal control; ^••^*P* < 0.01 and ^•••^*P* < 0.001, compared to diabetic control; °P <0.05, compared to MET; N-GH, normal-GH of 250 mg/kg; N-MET, normal-MET of 70 mg/kg; N-(GH + MET), GH plus MET in normal rats; D-GH, GH of 250 mg/kg in diabetic rats; D-MET, MET of 70 mg/kg in diabetic rats; and D-(GH + MET), GH plus MET in diabetic rats.

**Figure 3:** Effect on SOD and catalase in HTH. Data are given as mean ±SEM, where ^∗∗^*P* < 0.01 and ^∗∗∗^*P* < 0.001 compared to normal control; ^••^*P* < 0.01 and ^•••^*P* < 0.001, compared to diabetic control; °P <0.05, compared to MET; N-GH, normal-GH of 250 mg/kg; N-MET, normal-MET of 70 mg/kg; N-(GH + MET), GH plus MET in normal rats; D-GH, GH of 250 mg/kg in diabetic rats; D-MET, MET of 70 mg/kg in diabetic rats; and D-(GH + MET), GH plus MET in diabetic rats.

**Figure 4:** Levels of thiobarbituric acid substances in different experimental groups. Data are given as mean ±SEM, where ^∗∗^*P* < 0.01 and ^∗∗∗^*P* < 0.001, compared to normal control; ^••^*P* < 0.01 and ^•••^*P* < 0.001, compared to diabetic control; °P <0.05, compared to MET; N-GH, normal-GH of 250 mg/kg; N-MET, normal-MET of 70 mg/kg; N-(GH + MET), GH plus MET in normal rats; D-GH, GH of 250 mg/kg in diabetic rats; D-MET, MET of 70 mg/kg in diabetic rats; and D-(GH + MET), GH plus MET in diabetic rats.

**Figure 5:** Effect on percentage recovery in HR and DT. Data are given as mean ±SEM, where ^∗∗^*P* < 0.01 and ^∗∗∗^*P* < 0.001, compared to normal control; ^••^*P* < 0.01 and ^•••^*P* < 0.001, compared to diabetic control; °P <0.05, compared to MET; N-GH, normal-GH of 250 mg/kg; N-MET, normal-MET of 70 mg/kg; N-(GH + MET), GH plus MET in normal rats; D-GH, GH of 250 mg/kg in diabetic rats; D-MET, MET of 70 mg/kg in diabetic rats; and D-(GH + MET), GH plus MET in diabetic rats.

**Figure 6:** Histopathological slides of myocardial tissue. (a) Normal myocardial structure with integrity of membrane in nondiabetic control (normal control group). (b) Normal cardiac structure was observed in a section of the garlic-treated group. (c) The size of the cardiocytes appears to be reduced in the group treated with MET in this section. When contrasted with muscle tissue, the collagen tissue seems to be larger. Throughout the muscle tissue, there are scattered mononuclear inflammatory infiltrations. (d) The heart architecture of the group treated with MET and RGH is intact in this section. (e) Diabetic control section showing heart muscle with fibrovascular septae in between. The heart muscle appears to be in good condition. Between the heart muscle fibers, there are a few dispersed mononuclear inflammatory cells. (f) The cardiac architecture of diabetic animals treated with GH is intact in this section. The cardiocytes are placed haphazardly in some regions. The cardiocytes appear to be of normal size. (g) A section of the group that received MET showed myocardium and endocardium made up of cardiac muscle with fibrovascular septae in between. Between the heart muscle fibers, dispersed mononuclear inflammatory cells can also be observed. (h) Normal cardiac structure observed in the garlic and MET-treated groups.

**Figure 7:** Histopathological studies of pancreatic tissue (long arrow shows centrally located *ß* cells and small arrow denotes peripherally positioned *a* cells). (a) The lobules of the pancreas are distinguished by septa of connective tissue in nondiabetic control group (normal control group). *ß* cells (80%) were present in the central islets, while *a* cells (20%) were mainly in the periphery. (b) The lobules of the pancreas are demarcated with the septum of connective tissue in the garlic-treated group in nondiabetic rats. Almost 70% is made up of central islet *ß* cells and 25% giant *a* cells in the periphery. (c) The lobule of the pancreas was divided by connective tissue septa in a section of the group treated with metformin (MET). The lobules are generally spherical Langerhans islets. Small *ß*-cell aggregates (70 percent, short arrow) with basophilic granules make up the heart of islet cells, while big *a* cells (25 percent, long arrow) make up the periphery. Thin-walled crowded capillaries intervene between these cells. (d) The lobules of the pancreas were demarcated clearly with septa of connective tissue in sections of the group treated with metformin and GH. *ß* cells make up 75% of the islets while 20% are *a* cells in the periphery. (e) Pancreatic lobules are divided by connective tissue septa in a diabetic control section. A large number of lobules have substantial patches of light-stained Langerhans islets. *ß* cells (60 percent, long arrow) with basophilic granules make up the heart of islet cells, while *a* cells (35 percent, short arrow) with eosinophilic granules make up the periphery. A few degraded beta cells can also be detected. (f) The lobules of the pancreas are distinguished by septa of connective tissue in a section of the garlic-treated group in diabetic rats. The *ß* cells make up 70% of islet cells while 25% of alpha cells are mainly located at the periphery. (g) The pancreatic lobules of animals treated with MET in diabetic rats have *ß* cells (70%) and 25% *a* cells in the periphery. (h) The center of islet cells in diabetic rats treated with MET and GH has 70% *ß* cells and 25% *a* cells in the periphery.

**Table 1:** Effect on body weight and blood sugar.

Groups	Body weight (g)			Blood glucose (mg/dl)		
	Baseline	At the end of four weeks	At the end of eight weeks	Baseline	At the end of eight weeks	72 hours after alloxan
Diabetic control	202.71 ± 6.2	218.32 ± 9.2	245.52 ± 8.2^c^	160 ± 1.7	193.23 ± 3.5^b^	329.28 ± 3.1^c^
D-GH	210.98 ± 8.3	224.41 ± 10.3	252.54 ± 11.1^c^	148 ± 2.4	185.67 ± 7.7^b^	312.56 ± 7.5^c^
D-MET	204.73 ± 10.5	222.21 ± 8.8	258.32 ± 9.7^c^	110 ± 1.5	153.23 ± 6.9^b^	321.56 ± 8.5^c^
D-(GH + MET)	210.45 ± 8.2	226.82 ± 7.2	260.43 ± 8.3^c^	122 ± 1.8	185.39 ± 8.5^b^	316.54 ± 10.6^c^

Data are given as mean ± SEM, where ^b^*P* < 0.01 and ^c^*P* < 0.001 when compared to baseline; D-GH, GH of 250 mg/kg in diabetic rats; D-MET, MET of 70 mg/kg in diabetic rats; and D-(GH + MET), GH plus MET in diabetic rats.

## Data Availability

The data are available on request to the corresponding author.
